The article "A new Frontier in electric load forecasting: The LSV/MOPA model optimized by modified orca predation algorithm" was retracted in 2026. Reasons: errors in the text; unreliable results or conclusions; concerns about the citations; concerns about the authorship.

# A new Frontier in electric load forecasting: The LSV/MOPA model optimized by modified orca predation algorithm

**DOI:** 10.1016/j.heliyon.2024.e24183

**Published:** 2024-01-12

**Authors:** Guanyu Yan, Jinyu Wang, Myo Thwin

**Affiliations:** a School of Electrical and Information Engineering, Northeast Petroleum University, Daqing, 163318, Heilongjiang, China; b Yangon Technological University, Myanmar; c College of Technical Engineering, The Islamic University, Najaf, Iraq

**Keywords:** Electric load forecasting, Hybrid technique, Support vector regression, Long short-term memory, Modified orca predation algorithm, South Korea, Efficiency of algorithm, Comparative performance

## Abstract

Electric load forecasting is a vital task for energy management and policy-making. However, it is also a challenging problem due to the complex and dynamic nature of electric load data. In this paper, a novel technique, called LSV/MOPA, has been proposed for electric load forecasting. The technique is a hybrid model that combines the advantages of Long Short-Term Memory (LSTM) and Support Vector Regression (SVR), two powerful artificial intelligence algorithms. The hybrid model is further optimized by a newly Modified Orca Predation Algorithm (MOPA), which enhances the forecasting accuracy and efficiency. The LSV/MOPA model has been applied to historical electric load data from South Korea, covering four regions and 20 years. The LSV/MOPA model has been compared with other state-of-the-art forecasting techniques, including SVR/FFA, LSTM/BO, LSTM-SVR, and CNN-LSTM. The results show that the LSV/MOPA model with minimum average mean absolute percentage deviation error, including 365 in northern region, 12.8 in southern region, 8.6 in central region, and 30.8 in eastern region, provides the best fitting and outperforms the other techniques in terms of the Mean Absolute Percentage Deviation (MAPD) index, achieving lower values for all regions and years. The LSV/MOPA model also exhibits faster convergence and better generalization than the other techniques. This study demonstrates the effectiveness and superiority of the LSV/MOPA model for electric load forecasting and suggests its potential applications in other sectors where accurate forecasting is crucial.

## 1 Introduction

Electric load forecasting is a critical activity in the energy industry since it aids in resource planning, supply-demand management, and the effective operation of power systems. For predicting load, conventional forecasting techniques like time series models have been extensively employed. However, new methods like LSTM (Long Short-Term Memory) and SVR (Support Vector Regression) have grown in favor as a result of advances in machine learning and deep learning techniques because of their capacity to recognize intricate patterns and nonlinear correlations in the data.

A method for supervised learning that may be used to solve regression problems is SVR. With respect to the idea of SVM, it builds a hyperplane optimizing the boundary among various classes or, about regression cases, minimizing the mistakes existing between the anticipated and actual values using a subset of training data called support vectors. Due to its capacity to manage high-dimensional data and nonlinear interactions, SVR has been effectively employed in a number of domains, including load forecasting.

The LSTM, on the other hand, is a special kind of RNN (Recurrent Neural Network) that is designed to have relationships, which are long-term in sequential data. If some components are included, such as a cell of memory as well as three gating mechanisms (forget, output gates, and input) that handle the information flow, it solves the vanishing gradient issue of conventional RNNs. In time series forecasting applications such as load forecasting, LSTM has shown great performance due to its ability to efficiently capture temporal relationships and manage variable-length input sequences.

Load prediction is necessary to the smooth running of the electricity system in South Korea, which is controlled by the Korea Electricity Exchange (KPX). For the best generation planning, system's stability, precise load estimations, and energy trading are crucial. In South Korea, conventional time series models like ARIMA and SARIMA are often employed for load forecasting [1]. However, machine learning and deep learning models like SVR and LSTM have become more popular as a result of the complexity of load patterns and the accessibility of enormous quantities of data.

To investigate the use of SVR and LSTM in load forecasting, several research works have been carried out. For example, Tang et al. [2] suggested a multi-layer bidirectional RNN version with respect to GRU and LSTM for employing two datasets that projecting short-term power load was confirmed. The experimental results demonstrated that the suggested strategy outperformed the winner of competition regarding accuracy when anticipating on the competition data of European Intelligent Technology Network. For the data of energy office in Chongqing, hourly peak loads of different types of load data were used to conduct experiments while considering differences in seasonal load. The designers individually forecasted the load of seasons and compared it with Long Short-Term Memory, SVR, and backpropagation styles. The comparison findings showed that the proposed method had a higher forecasting accuracy than the adopted models.

El-Hendawi and Zhanle Wang [3] proposed an entire method of complete wavelet packet change and networks of nerves for predicting short-term load. This method, called the full wavelet neural network approach, involved using the complete wavelet packet change style to fall apart the profile of load and different attributes into several constituents with various frequencies, which were then utilized to practice the networks of nerves. To carry out load prediction, the full wavelet packet transform version fell apart attributes into various constituents that affected the trained networks of nerves, and the production of the networks were shaped as the load, which had been forecasted. The suggested approach was employed for predicting load in the electric store in Canada. The results from modelling showed that the suggested method reduced the MAPE (Mean Absolute Percentage Error) by 20 % compared to the strategies of conventional NNs. Utilities and system operators could use the proposed approach to anticipate energy usage with high meticulousness, which was really popular for operation of power system, integration of renewable energy and management of demand-side.

Oreshkin et al. [4] proposed the problem of mid-term electricity load forecasting, as an essential issue for energy process planning and operation, in addition to maintaining future agreements in unregulated markets for energy. They proposed a model in which network of nerves were really deep in light of the deep architecture of nerves, which proved to be effective at solving this forecasting problem. The model had a potent expression to deal with chaotic random prediction issues for time series with strong random fluctuations, trends, and volatility. Additionally, it was straightforward to implement and train, required no preprocessing of sign and fitted with a technique to reduce prediction bias. The authors conducted an empirical study and compared their approach to ten strategies, comprising machine learning, hybrid strategies, and classical statistical strategies, using 35 monthly demand time of energy series for different countries in Europe. The findings of the research showed that the suggested NN (neural network) outperformed all opponents regarding both precision and bias of prediction. The code used in the study is available on GitHub.

Yotto et al. [5] evaluated 3 strategies of an approach utilized in ANN (Artificial Neural Networks) for predicting energy usage that was the MLP (Multilayer Perceptron) using return propagation. To verify consistent and meticulous anticipation, an assessment method utilizing R (correlation coefficient) and MSE (Mean Square Error) was used. The findings indicated that the Bayesian regulating kind of the MLP (Multi-layer Perceptron) provided data that were very near original data while learning and practicing these strategies. The verified model has low anticipating deviations and excellent generalization properties.

Haydar et al. [6] proposed a framework for energy load anticipation that involved selection of attribute, extraction, as well as regression. XGB (Extreme Gradient Boosting) and RF (Random Forest) were used in the attribute selection phase to ascertain the value of each attribute. RFE (Recursive Feature Elimination) was applied to remove superfluous attributes in the attribute extraction method. An ESVM (Enhanced Support Vector Machine) and an ECNN (Enhanced Convolutional Neural Network) were proposed for the regression constituent, using hyperparameters set with the RS (Random Search) strategy. The effectiveness of the suggested methods was demonstrated through a juxtaposition with state-of-the-art approaches and statistical analyses. The suggested strategies ESVM and ECNN achieved higher precision of 98.7 % and 98.83 %, respectively, with respect to findings that are simulated.

These studies showed how useful SVR and LSTM models may be for load forecasting in South Korea. These models are suited for addressing the complicated load patterns seen in the nation because they can capture nonlinear connections and temporal dependencies in the data. It is crucial to remember that the efficiency of the models may differ with respect to the particular set of data, input attributes, and model setup.

SVR and LSTM models have shown promise for load forecasting in South Korea, in conclusion. These models might promote effective power system operation and increase the precision of load projections. To fully realize the promise of these models and handle the unique difficulties and needs of load forecasting in South Korea, more study and development in this field are required.

The research work presented in this study makes several significant contributions to the field of electric load forecasting. These contributions can be summarized as follows:

Development of the LSV/MOPA Model: The main advantage of this study is the development of the LSV/MOPA style, which combines SVR (Support Vector Regression) and LSTM (Long Short-Term Memory) techniques. This hybrid style is further enhanced by a newly Modified Orca Predation Algorithm (MOPA). The integration of these techniques and algorithms creates a novel and powerful forecasting model that outperforms other existing methods.

Improved Accuracy and Efficiency: The LSV/MOPA model demonstrates superior execution regarding efficacy and precision juxtaposed to other recent techniques. By leveraging the strengths of SVR and LSTM and optimizing the model using MOPA, the research work achieves more precise and reliable electric load forecasts. This improvement in accuracy and efficiency is crucial for policy-making and efficient management of electricity.

Comparative Analysis: The research work includes a comparative analysis of the LSV/MOPA model with other contemporary forecasting techniques. This analysis provides empirical evidence of the model's superiority and establishes its competitive edge in the field. By showcasing the comparative performance of the LSV/MOPA model, the research work contributes to the evaluation and selection of the most effective forecasting methods.

Implications for Energy Management and Policy-making: The outcomes of this research have some implications, which are really significant for electricity management as well as policy-making. Accurate electric load forecasting is crucial for optimizing resource allocation, planning energy generation, and ensuring grid's stability. The LSV/MOPA model's improved accuracy and efficiency can contribute to more effective decision-making processes in these domains, leading to enhanced energy management strategies and policies.

In general, the research work's contributions lie in the development of the LSV/MOPA model, its superior performance compared to other techniques, the practical application to South Korean data, and the implications for energy management and policy-making. These contributions advance the field of electric load forecasting and open the door to more precise and effective predicting techniques with broader applications in the energy industry. Therefore, the main contributions and innovations of this paper are as follows.

− A novel hybrid model, called LSV/MOPA, has been developed that integrates LSTM and SVR, two powerful AI algorithms, for electric load forecasting. The hybrid model can capture the nonlinear, nonstationary, and stochastic characteristics of electric load data and handle multivariate as well as sequential data, making it suitable for various regions and time scales.
− New optimization algorithm, called MOPA, has been designed that modifies the original Orca Predation Algorithm (OPA) by incorporating the Lévy flight mechanism, which improves the exploration and exploitation abilities of the algorithm. The MOPA algorithm can optimize the hyperparameters of the LSTM model, the kernel function, and its parameters of the SVR model, as well as the weights and biases of the hybrid model, making it more accurate and efficient.
− The LSV/MOPA model has been applied to historical electric load data from South Korea, covering four regions and 20 years. The LSV/MOPA model has been compared with other state-of-the-art forecasting techniques, such as SVR/FFA, LSTM/BO, LSTM-SVR, and CNN-LSTM. The results show that the LSV/MOPA model outperforms the other techniques in terms of the Mean Absolute Percentage Deviation (MAPD) index, achieving lower values for all regions and years. The LSV/MOPA model also exhibits faster convergence and better generalization than the other techniques.
− The effectiveness and superiority of the LSV/MOPA model has been demonstrated for electric load forecasting. Moreover, the efficiency and dominance of the model suggests its potential applications in other sectors where accurate forecasting is crucial. The implications and limitations of the research will also be discussed, and some directions for future work will be provided.

## 2 SVR/LSTM model

SVR and LSTM have widely utilized machine learning methodologies to predict time series. SVR has been regarded as a regression analysis strategy, which employs Support Vector Machines to forecast continuous variables. On contrary, LSTM (Long-Short-Term Memory) has been known as a kind of RNN (Recurrent Neural Network) that is known for its proficiency in modeling sequential data.

The integration of LSTM (Long-Short-Term Memory) and SVR (Support Vector Regression) techniques has the potential to enhance the precision of forecasting. This is because SVR is adept at capturing the linear associations in the data, while LSTM is proficient at capturing the non-linear associations and enduring dependencies.

The optimization of the model can be achieved through the utilization of a modified technique known as the balanced Orca predation algorithm. The algorithm in question draws inspiration from the hunting patterns exhibited by orcas, a species renowned for their adeptness at coordinated and harmonious hunting techniques. The algorithm known as balanced Orca predation operates by achieving equilibrium in exploitation and the exploration of the space which should be searched [7]. The methodology employed involves a population-centric strategy, whereby a group of potential solutions (or individuals) undergo assessment and iterative refinement across numerous generations.

The algorithm assesses the fitness of every member in a given generation by utilizing a fitness function that gauges the precision of the SVR-LSTM model. Subsequently, the algorithm proceeds to choose the most optimal candidates for procreation, entailing the amalgamation of genetic components from two distinct individuals to generate a novel progeny.

The algorithm incorporates a mutation operator that stochastically alters the genetic formation of an individual, thereby introducing novel variations within the population.

The utilization of the balanced Orca predation algorithm in optimizing the SVR-LSTM model has the potential to enhance its precision and resilience, thereby increasing its efficacy in time series forecasting endeavors. Fig. (1) illustrates a schema of an SVR model.

**Fig. 1:** Schema of an SVR

In the following, the utilized materials in this study are explained in details.

### 2.1 SVR

The SVR (Support Vector Regression) technique has been known as a form of regression analysis that employs SVMs (Support Vector Machine) to forecast continuous variables. The method exhibits notable efficacy in handling datasets that feature intricate nonlinear associations between the input and output variables.

The fundamental concept underlying Support Vector Regression is to identify a hyperplane that optimizes the distance between the projected outcomes and the factual outcomes. The margin can be characterized as the distance between the hyperplane and the closest vectors of support in space, corresponding to the data points that are in closest proximity to the hyperplane [8]. The stages of an SVR involves the following steps:

The process of data preprocessing is undertaken to ensure that the input data is appropriately formatted for utilization by the Support Vector Regression (SVR) algorithm. The process may entail the adjustment of data scaling, the elimination of outliers, and the management of missing values.

The process of training model involves iteratively adjusting the parameters of a machine learning algorithm to optimize its performance on the SVR (Support Vector Regression) algorithm that has been trained on preprocessed data with the objective of identifying the hyperplane that maximizes the margin [9]. The mathematical construct known as the hyperplane is established through the specification of a collection of weights (w) and a bias term (b).

In the process of model evaluation, the SVR (Support Vector Regression) system that is trained is subjected to assessment using an independent test dataset in order to gauge its efficacy. This may entail the computation of metrics, such as the MSE (Mean Squared Error) or the MAE (Mean Absolute Error) [10].

The Support Vector Regression (SVR) algorithm possesses multiple parameters that can be adjusted to enhance its overall performance [11]. The aforementioned items encompass:

The kernel function is a mathematical tool utilized for mapping the input data onto a space in a higher dimension, thereby facilitating the identification of a hyperplane that can effectively separate the data [12]. The kernel functions that are frequently employed in various machine learning algorithms comprise linear, polynomial, and Radial Basis Function (RBF).

The parameter of regularization (C) is responsible for regulating the balance between the maximization of the margin and the minimization of the error on the training data. A rise in the value of C will result in a decrease in the margin's width and an increase in the model's complexity, whereas a decrease in the value of C will lead to an enhancement in the margin's width and a decrease in the model's complexity.

The parameter denoted by epsilon (ε) establishes the magnitude of the zone that is insensitive to deviations of predicted values from the actual ones. Data points falling within this zone are deemed to be accurately predicted and do not make any contribution to the overall error.

The Support Vector Regression (SVR) algorithm has the potential to be mathematically defined as the resolution of a forced optimization issue, which can be represented as [equation (1)]:

(1) $$f=\min\frac{1}{2}{\left\|w\right\|}^{2}+C\sum_{i=1}^{n}\left(\varepsilon_{i}-\varepsilon_{i^{*}}\;\right)\text{.}$$

subject to [equations (1), (2), (3), (4)]:

(2) $$y_{i}-w^{T}x_{i}-b\leq \varepsilon_{i}\text{,}$$

(3) $$w^{T}x_{i}+b-y_{i}\leq \varepsilon_{i}^{*}\text{,}$$

(4) $$\varepsilon_{i},\varepsilon_{i}^{*}\geq 0,i=1,2,\ldots ,n\text{.}$$

The aforementioned equation involves the input vector $x_{i}$, its corresponding output value $y_{i}$, the upper and lower bounds of the epsilon-insensitive zone represented by $\varepsilon_{i}$ and $\varepsilon_{i}^{*}$, respectively, and the regularization parameter denoted by C.

The kernel trick is a method that can be employed to expand the utilization of SVR (Support Vector Regression) to non-linear functions. The utilization of the kernel trick enables the implicit mapping of input data into a feature space of higher dimensionality, thereby facilitating the identification of linear relationships. The utilization of Support Vector Regression (SVR) allows for the identification and analysis of non-linear patterns present within the dataset.

The kernel trick is a technique that entails substitution of the dot product between input vectors ($x_{i}$ and $x_{j}$) with a kernel function. The kernel function is responsible for computing the similarity or distance between the vectors in the higher-dimensional feature space. The revised version of Support Vector Regression (SVR) utilizing the kernel method can be represented in the subsequent manner [equation (5)]:

(5) $$f=\min\frac{1}{2}\times K\left(x_{i},x_{j}\right)+C\sum_{i=1}^{n}\left(\varepsilon_{i}-\varepsilon_{i^{*}}\;\right)\text{.}$$

subject to [equations (6), (7), (8), (9)]:

(6) $$\sum \left(\alpha_{i}-\alpha_{i}^{*}\;\right)=0\text{,}$$

(7) $$0\leq \alpha_{i},\alpha_{i}^{*}<C\text{,}$$

(8) $$y_{i}-\sum \left(\alpha_{i}-\alpha_{i}^{*}\;\right)\times K\left(x_{i},x_{j}\right)-b\leq \varepsilon_{i}\text{,}$$

(9) $$\sum \left(\alpha_{i}-\alpha_{i}^{*}\;\right)\times K\left(x_{i},x_{j}\right)-y_{i}\leq \varepsilon_{i}^{*}\text{.}$$

The present formulation involves the utilization of $K\left(x_{i},x_{j}\right)$ as the kernel function, which is responsible for computing the similarity or distance between the input vectors $x_{j}$ and $x_{i}$ within the attribute space of higher dimensionality. The kernel function determination has been considered to be contingent upon the particular problem at hand and the inherent attributes of the dataset. Here, Polynomial Kernel has been used.

The Polynomial Kernel can be represented as follows [equation (10)]:

(10) $$K\left(x_{i},x_{j}\right)={\left(\gamma x_{i}^{T}x_{j}+r\right)}^{d}\text{.}$$

where, γ, r, and d are constants.

The utilization of the polynomial kernel facilitates the capture of polynomial associations among the input variables.

Support Vector Regression (SVR) is capable of efficiently capturing arbitrary associations among the output and input elements through the utilization of suitable kernel functions. The utilization of the kernel trick enables Support Vector Regression (SVR) to function implicitly in a feature space of higher dimensionality, without the need for explicit computation of the transformed feature vectors, thereby enhancing its computational efficiency.

### 2.2 LSTM

The LSTM (Long Short-Term Memory) is a special kind of architecture for RNNs, which has been developed to address the issue of the vanishing gradient and to effectively model long-term dependencies in sequential data. This is accomplished through the utilization of a memory cell and multiple gating mechanisms that regulate the transmission of data. The LSTM architecture comprises a number of essential components, which are explained in the following.

The rudimentary parameter of an LSTM is the memory cell. The network is enabled to retain and retrieve data across extended sequences. At each time step, the memory cell is responsible for updating both a hidden state ($h_{t}$) and a cell state ($c_{t}$).

According to Gates, LSTM versions have been equipped with three distinct gates, namely the gate of input ($i_{t}$), the gate of forget ($f_{t}$), and the gate of output ($o_{t}$), which have been regarded responsible for regulating the flow of information. The function of these gates pertains to the selective modification and retrieval of data from the cell of memory.

The responsibility of regulating the amount of novel information is on the Input Gate ($i_{t}$), which must be stored in the cell of memory. The function receives two inputs, including the previous state that is hidden ($h_{t-1})$ and the present input ($x_{t}$), and generates an output that ranges from 0 to 1.

The forget gate ($f_{t}$) regulates the degree to which the preceding cell state ($c_{t-1}$) is to be disregarded. The function accepts the previous state, which is hidden, and the present input as inputs; in addition, it generates an output within the range of 0 and 1.

The responsibility of controlling the quantity of data is on the Gate of Output ($o_{t}$), which is released from the cell of memory.

Updating state of the cell is contingent upon the input gate, the antecedent state of cell, and forget gate. The gates of input and forget are two crucial components of the LSTM style. The former has responsibility for determining how much of the prior cell state should be kept, while the latter is responsible for determining the extent to which new information should be incorporated into the state of cell.

The computation of the state, which is hidden ($h_{t}$), is contingent upon the updated cell state and the output gate. The concealed state conveys pertinent data from the recollection unit to the subsequent temporal phase.

Regarding its parameters, an LSTM possesses the following details:

LSTMs are equipped with weight matrices that correspond to the input, hidden state, and bias terms linked to update of the cell state, output gate, forget gate, and the input gate.

LSTMs are equipped with bias terms that are linked to update of the cell state, output gate, forget gate, and the input gate.

The activation functions employed in LSTMs are typically the sigmoid function for the gates of the output, forget, input, and the function of hyperbolic tangent (tanh) for updating the state of hidden cell.

Throughout the training phase, the LSTM parameters are acquired via the Backpropagation Through Time (BPTT) technique, wherein the gradients are calculated and, subsequently, utilized to modify the weights and biases.

The LSTM models have gained significant traction in diverse domains, such as processing of natural language, recognition of speech, and analysis of time series. This is attributed to their remarkable capacity to capture long-term dependencies and effectively processing the sequential data. Fig. (2) illustrates a schema of a Long Short-Term Memory model.

**Fig. 2:** Block diagram of an LSTM model.

The LSTM (Long Short-Term Memory) structure comprises multiple layers, encompassing the layer of input and output and LSTM. The mathematical equations will be examined pertaining to each of these layers.

The first layer, which has been known to be the input layer, is responsible for receiving the input sequence during each individual time step. The input at a given time step t can be represented as $x_{t}$. The input layer is primarily responsible for transmitting the input to the LSTM layers without performing any computational operations.

The LSTM layer is a kind of RNN layer, which has been created to serve as the fundamental element of the Long Short-Term Memory framework. The system is comprised of multiple constituents, such as the cell of memory, forget gate, input gate, hidden state, and output gate.

The memory cell is a fundamental element of computer memory, which has the responsibility for retrieving and storing data. The updated equations for the memory cell are given below [equation (11), (12), (13), (14), (15)]:

(11) $$i_{t}=\sigma \left(W_{i}*x_{t}+U_{i}*h_{t-1}+b_{i}\right)\;\left(input\;gate\right)\text{,}$$

(12) $$f_{t}=\sigma \left(W_{f}*x_{t}+U_{f}*h_{t-1}+b_{f}\right)\;\left(forget\;gate\right)\text{,}$$

(13) $$o_{t}=\sigma \left(W_{o}*x_{t}+U_{o}*h_{t-1}+b_{o}\right)\;\left(output\;gate\right)\text{,}$$

(14) $$g_{t}=\tanh\left(W_{g}*x_{t}+U_{g}*h_{t-1}+b_{g}\right)\;\left(cell\;input\right)\text{,}$$

(15) $$c_{t}=f_{t}*c_{t-1}+i_{t}*g_{t}\;\left(cell\;state\;update\right)\text{.}$$

where, the sigmoid activation function denoted by σ(.), the hyperbolic tangent activation function denoted by tanh(.), and matrix multiplication denoted by *.

Hidden state is the next layer of the LSTM. The notation $h_{t}$ is utilized to represent the hidden state during the $t^{th}$ time step. The transmission of pertinent data from the memory cell to the subsequent time step is accomplished through the utilization of the subsequent equations [equation (16)]:

(16) $$h_{t}=o_{t}*\tanh\left(c_{t}\right)\;\left(hidden\;state\right)\text{.}$$

The final layer of a neural network that has known to be the output layer has the duty to produce the predictions of network. The output layer takes the hidden state $h_{t}$ at the final time step. The layer utilized may vary depending on the specific task, and may include a fully connected layer or another suitable option. The final output is generated by the application of an activation function to a linear transformation carried out by the output layer.

equation (17) is a mathematical expression that involves the variable y, which is a function of the product between the weight matrix $W_{y}$ and the hidden state $h_{t}$, added to the bias term $b_{y}$. The given equation utilizes the activation function f(.) to produce the final output as follows:

(17) $$y=f\left(W_{y}*h_{t}+b_{y}\right)\text{.}$$

The aforementioned equation involves the utilization of an activation function, denoted as f(.), which is applied in an element-wise manner to the vector $W_{y}*h_{t}+b_{y}$.

### 2.3 SVR/LSTM model

SVR (Support Vector Regression) is an algorithm of machine learning that has been widely employed for analysis of regression. The methodology influences the foundational concepts of SVM, a widely adopted classification algorithm, and adapts them to address predictive regression challenges. SVR (Support Vector Regression) is a valuable tool in the analysis of data with a high number of dimensions.

Conversely, the LSTM (Long Short-Term Memory) is a variant of RNN that exhibits the ability to acquire and retain information over extended data sequences, thereby rendering it a potent tool for analyzing time series data. The ability to achieve dependencies in long-term in sequencing data is particularly advantageous for achieving precise predictions in time series forecasting.

The Support Vector Regression (SVR) component has demonstrated efficacy in effectively managing data of high-dimensional, whereas the LSTM (Long Short-Term Memory) component has exhibited the ability to achieve dependencies in long-term present in the data. The combination of the aforementioned models has the potential to furnish more precise prognostications of load demand patterns in a microgrid (MG) across both abbreviated and protracted timeframes. The hybrid structure of the LSTM/SVR model is illustrated in Fig. (3).

**Fig. 3:** Hybrid structure of the SVR/LSTM model.

The use of periodic features as inputs for the SVR 1s (Support Vector Regression) is depicted in the figure, which enables the computation of a sequence of preliminary load values. The present study utilizes the latest recorded data point as a time series. The utilization of anomalous characteristics as inputs for SVR, specifically SVR 2, and LSTM models includes the incorporation of steady and time series as exemplars.

The variables Oy2 and Oy1 represent the results obtained from the LSTM model and SVR model, respectively. The ultimate output of the LSTM and SVR model could be predicted by the amalgamation of Oy1 and Oy2, as stated in Ref. [13].

## 3 The balanced orca predation algorithm

### 3.1 Preliminary steps

This section will explicate the methodologies that are imperative for developing the suggested approach. Elaborate accounts of the mathematical model of the OBL notion, the OPA (Orca Predation Algorithm), and the Lévy flight mechanism are comprehensively delineated.

### 3.2 Orca predation algorithm (OPA)

Yuxin et al. [14] have innovatively designed a novel nature-inspired optimization technique known as OPA, which emulates the attacking patterns of orcas; moreover, it dissects the patterns into distinct phases: encircling, attacking, and driving. Orca predation algorithm incorporates diverse strategies for driving and encircling, wherein parameter modifications are geared towards accomplishing a harmonious balance within exploitation and exploration. In the assaulting phase, OPA identifies the optimal solution while concurrently preserving the heterogeneity of particles through the consideration of the positions of numerous top-performing orcas and a selection cohort of randomly chosen orcas.

The OPA algorithm's mathematical definitions are presented below.

1. The advancement of a community of orcas entails the utilization of a cluster of $N_{n}$ orcas in the OPA, wherein they are depicted in one, two, three, or even higher dimensions. This depiction is illustrated in equation below [equation (18)]:

(18) $$Z=\left[z_{1},z_{2},z_{3},\ldots ,{zN}_{n}\right]=\left[\begin{array}{c} \begin{array}{cc} Z_{1,1} & \ldots \end{array}\;\begin{array}{ccc} Z_{1,2} & \ldots & Z_{1,\dim} \end{array}\\ \begin{array}{cc} \vdots & \ddots \end{array}\;\begin{array}{ccc} \vdots & \ddots & \vdots \end{array}\\ \begin{array}{cc} Z_{2,1} & \ldots \end{array}\;\begin{array}{ccc} Z_{2,2} & \ldots & Z_{2,\dim} \end{array}\\ \begin{array}{cc} \vdots & \ddots \end{array}\;\begin{array}{ccc} \vdots & \ddots & \vdots \end{array}\\ \begin{array}{cc} Z_{N_{n},1} & \ldots \end{array}\;\begin{array}{ccc} Z_{N_{n},2} & \ldots & Z_{N_{n},\dim} \end{array} \end{array}\right]\text{.}$$

where, Z represents the population of the orca in the potential solutions. The location of the $N^{th}$ orca member is denoted by ${zN}_{n}$, while the location of the $\dim^{th}$ dimension of the $N^{th}$ population is denoted by ${zN}_{n}$ and Dim.

2. The pursuit stage comprises two different steps, namely driving and encircling. To regulate the likelihood of these two stages being executed in isolation, $g_{1}$ is employed. This constant takes on values within the interval [0,1], and a random value is generated within this same interval. If the generated value exceeds $g_{1}$, the process of driving is executed; otherwise, the process of encircling is carried out.
3. The process of driving, to stop the orca deviating from the intended course, necessitates the regulation of the central position of the orca group, ensuring its proximity to the prey. equations (19), (20) depict the orca's velocity and its pertinent position:

(19) $$V_{\text{pursuit},1,i}^{t}=a\times \left(d\times z_{best}^{t}-P\times \left(b\times K^{t}+c\times z_{i}^{t}\right)\right)\text{,}$$

(20) $$V_{\text{pursuit},2,i}^{t}=e\times z_{best}^{t}-z_{i}^{t}\text{.}$$

where, t represents the quantity of iterations, $V_{\text{pursuit},1,i}^{t}$ signifies the pursuing pace after opting the first pursuing stage, and $V_{\text{pursuit},2,i}^{t}$ denotes the pursuing speed after electing the second pursuing stage. Furthermore, a, b, and d are random elements between [0, 1]. Similarly, e is a haphazard value within the range of [0, 2]. P is tantamount to 2, and h is a variable within the range of [0, 1], which is utilized for picking the pursuing procedure. Meanwhile, K represents the location in which the orcas are usually located, which has been demonstrated in equations (21), (22):

(21) $$K=\frac{\sum_{i=1}^{N_{n}}z_{i}^{t}}{N_{n}}\text{,}$$

(22) c=1−b.

There exist two distinct pursuing techniques predicated on the number of orcas in the population. In the occasion of a substantial orca population, that is, when the random variable exceeds the threshold value h, the initial approach is executed. Conversely, if the random variable is less than h, the secondary approach is implemented, as demonstrated in equation (23):

(23) $$\left\{ \begin{array}{c} z_{\text{pursuit},1,i}^{t}=z_{i}^{t}+V_{\text{pursuit},1,i}^{t}\;if\;\text{rand}>h\;\\ z_{\text{pursuit},2,i}^{t}=z_{i}^{t}+V_{\text{pursuit},2,i}^{t}\;if\;\text{rand}\leq h\; \end{array}\right.\text{.}$$

4. In this step, the orcas engage in a maneuver known as "encircling of prey". This involves utilizing the positional data of three selected orcas at random, which can be mathematically expressed as follows [equation (24), (25)]:

(24) $$z_{\text{pursuit},3,i,w}^{t}=z_{d1,w}^{t}+u\times \left(z_{d2,w}^{t}-z_{d3,w}^{t}\right)\text{,}$$

(25) $$u=2\times \left(randn-\frac{1}{2}\right)\times \frac{Maxrep-t}{Maxrep}\text{.}$$

where, Maxrep represents the maximum repetition quantities, and d1, d2, and d3 determine the selection of three randomly certain orcas from the total population of $N_{n}$ orcas, where it is required that d1 is not equal to d2 and d3. The scenario of selecting the third pursuing procedure is illustrated by $z_{\text{pursuit},3,i,w}^{t}$.

5. The state of orcas undergoes modifications across the encircling stage. These circumstances are governed in accordance with the succeeding formulaic equations [equation (26)]:

(26) $$\left\{ \begin{array}{c} z_{\text{pursuit},i}^{t}=z_{\text{pursuit},i}^{t}\;if\;p\left(z_{\text{pursuit},i}^{t}\right)<p\left(z_{i}^{t}\right)\\ z_{\text{pursuit},i}^{t}=z_{i}^{t}\;if\;p\left(z_{\text{pursuit},i}^{t}\right)\geq p\left(z_{i}^{t}\right) \end{array}\right.\text{.}$$

where, $p\left(z_{i}^{t}\right)$ indicates the fitness function associated with $z_{i}^{t}$, and $p\left(z_{\text{pursuit},i}^{t}\right)$ represents the fitness function linked to $z_{\text{pursuit},i}^{t}$.

6. During hunting the prey, the four most optimal assaulting positions, which are occupied by four orcas, are delineated in a circular formation. The subsequent equations are employed to ascertain the orcas' velocity and spatial coordinates throughout the assault process [equations (27), (28), (29)].

(27) $$V_{\text{assault},1,i}^{t}=0.25\times \left(z_{1}^{t}+z_{2}^{t}+z_{3}^{t}+z_{4}^{t}\right)-z_{pursuit,i}^{t}\text{,}$$

(28) $$V_{\text{assault},2,i}^{t}=\frac{1}{3}\times \left(z_{pursuit,d1}^{t}+z_{pursuit,d2}^{t}+z_{pursuit,d3}^{t}\right)-z_{i}^{t}\text{,}$$

(29) $$z_{\text{assault},i}^{t}=z_{pursuit,i}^{t}+f_{1}\times V_{\text{assault},1,i}^{t}+f_{2}\times V_{\text{assault},2,i}^{t}\text{.}$$

where, $V_{\text{assault},1,i}^{t}$ and $V_{\text{assault},2,i}^{t}$ denote the velocity vectors, and $z_{1}^{t}$, $z_{2}^{t}$ , $z_{3}^{t}$ and $z_{4}^{t}$ correspond to the four orcas in optimal location. d1, d2, and d3 represent three orcas randomly selected from $N_{n}$ throughout the pursuit step, where d1 ≠ d2 ≠ d3, and $z_{\text{assault},i}^{t}$ designates the location that is subsequent to the assault process. Additionally, $f_{1}$ denotes a stochastic variable sampled from the range [0, 2], and $f_{2}$ is a number being chosen randomly within [-2.5, 2.5].

7. During the phase of assault, the alterations of location occur. The precise location of the orca is ascertained through the identification of the lower boundary, denoted as $l_{l}$. This identification can be achieved following the provided outline [equation (30)]:

(30) $$if\;p\left(z_{\text{pursuit},i}^{t}\right)<p\left(z_{i}^{t}\right)\text{,}$$

$$Z_{i}^{t+1}=z_{\text{assault},i}^{t}\text{,}$$

Else Q=randn,

For w from 1 to D,

If Q<g2,

$$z_{j,w}^{t+1}=l_{l}\left(w\right)\text{,}$$

Else

$$z_{j,w}^{t+1}=z_{\text{pursuit},i,w}^{t+1}\text{.}$$

End.

End.

End

where, g2 denotes a numerical quantity that belongs to the interval encompassing values between zero and one.

In conclusion, the OPA algorithm's execution can be illustrated by the subsequent stages.

Stage 1 The orca populations and their corresponding parameters are initialized by setting the population's size, $N_{n}$, dimension, Dim, maximum number of repetitions, Maxrep, selection probabilities g1 and g2, lower limit, $l_{l}$, and upper limit, $u_{l}$. The orcas are randomly assigned positions within the range of $l_{l}$ and $u_{l}$.

Stage 2 The function value of every orca has been determined, and the best possible fitness has been identified as $Z_{best}$.

Stage 3 The location of the orca group is currently undergoing renews throughout the pursuing phase. At this phase, the decision on to encircle or drive the prey is dependent on the choosing factor g1, which is determined by the orcas. The locations are renewed according to Eqs. (19), (20), (21), (22), (23), (24), (25), (26).

Stage 4 The orcas modified their locations during the assaulting phase. These locations are renovated through the utilization of Eqs. (27), (28), (29), and substituted by $l_{l}$ subsequently, as demonstrated in Eq. (30).

Stage 5 Following the assaulting approach, the novel population will be greater to form a novel group.

Stage 6 The ending standards for the given procedure is met when the present number of repetitions surpasses the maximum permissible value. In the occasion that the desired output is not achieved, the second step of the earlier outlined processes will be reiterated.

### 3.3 The balanced orca predation algorithm

The Orca Predation Algorithm is a metaheuristic strategy that is stemmed from the hunting manner of orcas. This approach employs the simulation of the group hunting behavior of orcas to address optimization problems. Nevertheless, the algorithm may encounter premature convergence and exhibit a sluggish convergence rate. In order to tackle the aforementioned concerns, it is possible to implement a modification known as Lévy flight to the algorithm [15]. The Lévy flight adaptation incorporates a stochastic process with a power-law probability distribution into the computational procedure. This enables the algorithm to efficiently explore the search space and evade local optima. The incorporation of Lévy flight modification into the search process enhances its diversity, potentially resulting in improved solutions. The utilization of the Lévy flight modification in the Orca Predation Algorithm offers certain benefits, which have been listed down in the following.

- Enhanced investigation of the search domain.
- Accelerated convergence rate.
- The search process has been enhanced by an increased level of diversity.
- More effective alternatives
- The mechanism of Lévy flight can be formulated in the following way [equation (31), (32), (33)]:

(31) $$Le\left(w\right)\approx \frac{1}{w^{1+\tau }}\text{,}$$

(32) $$w=\frac{A}{{\left|B\right|}^{1/\tau }}\text{,}$$

(33) $$\sigma^{2}={\left(\frac{\Gamma \left(1+\tau \right)}{\tau \Gamma \left(\left(1+\tau \right)/2\right)}\frac{\sin\;\left(\pi \tau /2\right)}{2^{\left(1+\tau \right)/2}}\right)}^{\frac{2}{\tau }}\text{.}$$

where, τ defines index of the Lévy flight, w signifies the size of step, Γ(.) determines function of the Gamma, 0<τ≤2, $A∼N\left(0,\sigma^{2}\right)$, $B∼N\left(0,\sigma^{2}\right)$, and $A/B∼N\left(0,\sigma^{2}\right)$ refer to the examples made by a Gaussian distribution with zero mean value and $\sigma^{2}$ variance. Here, τ=3/2 [16], respectively.

Based on the defined mechanism, the new updated equation for the clan and the separating operators are as follows [equation (34)]:

(34) $$z_{new}^{t}=\underline{z^{t}}+\left(1+\bar{z^{t}}-\underline{z^{t}}\right)\times \text{Le}\left(\delta \right)\text{.}$$

where, $z_{new}^{t}$ defines the new updated position for the predator j.

Furthermore, to ensure the selection of optimal candidates of solution, only candidates that are fitter are retained, i.e. [equation (35)].

(35) $$z_{new}^{t}=\left\{ \begin{array}{c} z_{new}^{t}\;F\left(z_{new}^{t}\right)>F\left(z_{\text{pursuit},3,i,w}^{t}\right)\\ z_{\text{pursuit},3,i,w}^{t}\;otherwise \end{array}\right.\text{.}$$

To verify the efficacy of the algorithm under consideration, some studies were carried out on a commonly used benchmark function. The experiments were conducted on a computer system with the specifications below: The processor in question is the Intel(R) Core(TM) i7-9700K, which operates at a clock speed of 3.60 GHz. The system's Random Access Memory (RAM) capacity is 64 gigabytes. The computer's operating system is Windows 10 Professional 64-bit. The utilized software in this study is MATLAB 2017b.

The utilized benchmark function comprised 12 distinct functions extracted from the “CEC-BC-2017 test suite”. These functions were selected to encompass a diverse range of optimization problem landscapes. The aforementioned functions are frequently employed within the realm of optimization for the purpose of evaluating the efficacy of novel algorithms. The outcomes of our suggested algorithm were compared with those of five contemporary metaheuristic algorithms, namely Tunicate Swarm Algorithm (TSA) [17], GSA (Gravitational Search Algorithm) [18], MVO (Multi-Verse Optimizer) [19], PIO (Pigeon-Inspired Optimization) algorithm [20], and SDO (Supply-Demand-Based Optimization) [21]. To ensure the reliability of the results, all benchmark functions were subjected to 25 runs in each algorithm. The assessment of each algorithm's efficacy was predicated on the optimal solution attained and the rate of convergence. The findings indicate that the algorithm that was proposed exhibited superior performance compared to other algorithms, with respect to both the quality of solutions and the speed of convergence. In the current study, Table 1 illustrates the variable's values that were used in different optimization strategies.

**Table 1:** variable values used in different optimization strategies.

Algorithm	Parameter	Value
TSA (Tunicate Swarm Algorithm) [17]	Agents of search	50
	$P_{\min}$	2
	$P_{\max}$	2
	Quantity of generations	200
GSA (Gravitational Search Algorithm) [18]	Agents of search	50
	Constant Gravitation	40
	Coefficient of alpha	10
	Quantity of generations	200
Multi-Verse Optimizer (MVO) [19]	$WEP_{\min}$	0.1
	$WEP_{\max}$	0.9
	Coefficient (P)	5
Pigeon-Inspired Optimization Algorithm (PIO) [20]	Number of pigeons	50
	Dimension of space	10
	Compass and map factor	0.1
	Operation limit of compass and map	100
	Operation limit of landmark	200
	Inertia factor (w)	1
	Self-confidence factor ($c_{1}$)	1.2
	Swarm confidence factor ($c_{2}$)	1.2
Supply-Demand-Based Optimization (SDO) [21]	Max Iteration	200
	Market Size	30
	Fun Index	1

Statistical methods, such as the Best, Mean, and StD (Standard Deviation) of the performance index values were employed to analyze the experimental results. The purpose of this analysis was to ascertain the mathematical excellence of the performance distinctions among the BOPA and the other algorithms. The outcomes were additionally depicted through a table to facilitate a more intuitive comprehension of the variations in performance. Table 2 provides a comparison of the results obtained from BOPA and various sophisticated algorithms.

**Table 2:** Comparison of the results obtained from BOPA and various sophisticated algorithms.

Function	indicator	TSA [17]	GSA [18]	MVO [19]	PIO [20]	SDO [21]	BOPA
F1	Best	0.00	147.78	0.00	2.10	0.00	0.00
	Mean	0.00	263.00	5.71	11.38	6.66	0.00
	StD	0.00	192.76	74.34	14.49	88.03	0.00
F2	Best	7.17	321.45	0.19	171.91	54.29	0.14
	Mean	96.99	1782.61	0.63	1090.47	0.06	0.02
	StD	45.59	1368.81	0.54	327.37	0.08	0.04
F3	Best	0.01	28.51	0.01	1.63	0.06	0.00
	Mean	0.04	38.80	0.11	12.61	0.13	0.00
	StD	0.01	10.68	0.26	10.70	0.27	0.00
F4	Best	0.14	4.97	0.0.5	9.15	0.09	0.00
	Mean	0.38	9.98	0.00	12.55	0.00	0.00
	StD	0.13	1.42	0.01	2.28	0.01	0.00
F5	Best	0.00	3.73	0.00	0.12	0.00	0.00
	Mean	0.01	5.82	0.00	1.81	0.00	0.00
	StD	0.00	1.87	0.00	1.15	0.00	0.00
F6	Best	0.00	0.12	0.00	1.76	0.00	0.00
	Mean	0.00	72.97	0.53	1.42	0.63	0.00
	StD	0.00	218.79	1.08	1.50	1.70	0.00
F7	Best	0.72	104.35	0.25	0.80	0.33	0.03
	Mean	1.14	290.93	12.31	12.29	13.76	0.04
	StD	0.21	81.60	13.69	10.62	21.64	0.02
F8	Best	11.96	29.73		133.35	6.09	11.37
	Mean	13.81	32.56	18.65	910.40	0.00	0.00
	StD	6.61	15.06	0.19	767.12	0.00	0.00
F9	Best	0.00	15.15	0.00	0.11	0.00	0.00
	Mean	0.00	35.10	0.12	2.57	0.19	0.00
	StD	0.00	8.79	3.47	1.82	4.08	0.00
F10	Best	3.24	67.95	3.86	32.87	5.32	1.44
	Mean	4.24	176.88	14.57	121.37	0.00	1.08
	StD	5.45	28.09	6.84	51.18	0.01	0.01
F11	Best	0.00	0.05	0.00	0.10	0.00	0.00
	Mean	0.01	0.17	0.00	0.47	0.00	0.00
	StD	0.00	0.13	0.00	0.10	0.00	0.00
F12	Best	0.00	0.00	0.00	0.00	0.00	0.00
	Mean	0.00	0.00	0.00	0.00	0.00	0.00
	StD	0.00	0.00	0.00	0.00	6.66	0.00

As can be observed from the results, the BOPA algorithm has demonstrated its superior accuracy and consistency by obtaining the lowest values of the Best, Mean, and StD indicators for most of the functions. Additionally, the BOPA algorithm has proven its capability to handle various types of optimization problems, including unimodal, multimodal, separable, and non-separable functions. The BOPA algorithm has significantly outperformed the other algorithms, particularly on the more complex and challenging functions F2, F4, F6, F8, F10, and F12. Furthermore, the results indicate that the BOPA algorithm has a faster convergence rate than the other algorithms, as it can reach the optimal or near-optimal solutions within fewer iterations. These findings demonstrate the effectiveness and superiority of the BOPA algorithm in solving optimization problems and suggest its potential applications in other domains that require optimization.

### 3.4 BOPA for selecting the hyper-parameter of LSTM

The accuracy and performance of LSTM have been significantly impacted by its parameters. The determination of hyper-parameters is crucial in the training of LSTM models. These hyper-parameters include batch size, the input length (L), maximum training epochs, and number of hidden layer units (H). By selecting an appropriate input for L, it is possible to eliminate extraneous input information and enhance its overall performance. The impact of batch size on convergence efficacy has been noted [22]. The variable H will have an impact on the fitting outcome. The number of epochs in an LSTM (Long Short-Term Memory) model can have an impact on its convergence rate and fitting performance. The issue of extensive computation presents itself, necessitating the use of intelligent algorithms to select appropriate parameters that strike a balance between efficacy of computation and forecasting precision. The current study provides the introduction of BOPA as a novel and effective approach for selecting optimal parameters of the LSTM. Fig. (4) depicts the flowchart of BOPA/LSTM.

**Fig. 4:** Flowchart of BOPA/LSTM

At the first stage, the data are separated in two groups of test sets and training sets. Then, parameters' setting and initializing the algorithm and LSTM network are set. Then the BOPA is applied to the network to minimize the network's fitness, i.e. [equation (36)]

(36) $$minimize\;MSE=\text{minimize}\;\frac{1}{T}\sum_{j=1}^{L}\sum_{i=1}^{M}e_{ij}^{2}\left(t\right)\text{.}$$

Here [equation (37)],

(37) $$e_{ij}\left(t\right)=d_{ij}\left(t\right)-y_{ii}\left(t\right)\text{.}$$

The network's desired output is represented by $d_{ij}\left(t\right)$, while the network output achievement is determined by the equation of $y_{ij}\left(t\right)$, i.e. [equation (38)],

(38) $$y_{ij}\left(t\right)=f\left(\sum w_{li}z_{ip}+w_{l0}\right)\text{.}$$

where, l=1,2,…,m.

The main goal of the current research is to use BOPA to minimize Eq. (36) by optimizing the decision variables of LSTM and implementing a more efficient training approach to overcome the limitations of the previous algorithms.

## 4 Data set description

The proposed BOPA/LSTM-SVR model exhibited remarkable efficiency when applied to regional electric load data for South Korea spanning from 2001 to 2020 [23]. In order to validate the system, the prediction findings were compared with other models of regression. To this end, relevant data were collected and is presented in Table 3. Generally, the findings depict that the BOPA/LSTM-SVR model outperforms competing regression models in terms of accuracy and reliability.

**Table 3:** Relevant data of load demand for South Korea from 2001 to 2020.

Year	Load values in the North Region (MW)	Load values in the central part Region (MW)	Load values in the South region (MW)	Load values in the East Region (MW)
2001	3538	1813	2422	272
2002	3673	1979	2496	277
2003	3902	2307	2644	298
2004	4446	2369	2836	292
2005	4400	2340	2979	293
2006	5163	2788	3322	326
2007	5895	2962	3501	356
2008	6470	3415	3805	377
2009	6994	3526	3973	386
2010	7763	3805	4406	393
2011	7701	4193	4698	414
2012	8502	4575	4953	448
2013	8931	4744	5342	457
2014	9550	4921	5502	475
2015	10,404	4633	5947	493
2016	10,869	5085	6519	513
2017	11,372	5211	6486	508
2018	11,792	5396	6468	547
2019	12,131	5383	6409	551
2020	13,074	5783	6954	570

The dataset comprises load data of regional electricity sourced from South Korea, covering a time frame of two decades, commencing in 2001 and concluding in 2020. The aforementioned data hold significant importance in comprehending the trends in electricity usage, thereby facilitating the formulation of energy policies and infrastructure development strategies. The dataset has been partitioned into two distinct subsets with the aim of constructing and evaluating predictive models. The two groups are datasets of the test and training. Each of the sets fulfills a distinct application within the process of developing and evaluating a model.

The data set of training has been considered to be the most extensive collection of data, encompassing a period of 14 years. The aim of this is to facilitate the training of the predictive style. The data are utilized by the model to acquire knowledge of patterns and correlations, which can subsequently be employed to forecast forthcoming electricity loads. The period spanning from 2001 to 2015 is regarded as the training dataset.

The test of dataset comprises data spanning within a period of six years. The purpose of this procedure is to assess the efficacy of a trained predictive style. The evaluation of the model's accuracy and adjustment of its parameters are performed by comparing its predictions to the actual data in the testing set, which is a common practice among researchers. The period spanning from 2016 to 2020 is regarded as the test of dataset.

## 5 Simulation results

### 5.1 Parameters' estimation based on the proposed BOPA/LSTM-SVR model

The BOPA/LSTM-SVR model is employed in the realm of electrical load forecasting within South Korea to anticipate electric loads across various regions throughout a designated time frame. The suggested style integrates the advantageous attributes of the LSTM, BOPA, and SVR methodologies.

The model utilizes the BOPA component to ascertain the most suitable SVR parameters, which include Lag (L), Horizon (H), batch size, and Epochs. The aforementioned parameters are of paramount importance in the process of model training and the parallel minimization of training error. Through the utilization of the BOPA algorithm, the model is able to methodically explore various parameter combinations, ultimately leading to an enhancement in the precision of forecasting.

Upon identification of the optimized-selected parameters, they are supposed the most appropriate variables for employment in the BOPA/LSTM-SVR model. The selection of these parameters is based on their capacity to decrease the training error, then improve the predictive capabilities of the style. The outcomes of the prediction for various areas by BOPA/LSTM-SVR model are presented in Table 4.

**Table 4:** Findings of the prediction for various areas by BOPA/LSTM-SVR model.

Regions	Variables				MAPD (%)
	L	H	Batchsize	Epochs	
East	55	18	19	35.49	2.39
South	33	36	35	24.05	1.22
Center	18	41	58	25.37	1.38
North	35	20	96	14.18	1.15

As indicated, Table 4 is likely a presentation of the outcomes of the forecast derived from diverse BOPA/LSTM-SVR model methodologies. The findings suggest that the BOPA/LSTM-SVR model has shown a notable level of precision and reliability in predicting the electric load for various regions, as seen by the low and similar values of the Mean Absolute Percentage Deviation (MAPD). The findings also indicate that the BOPA/LSTM-SVR model has been successfully adjusted to the unique features and patterns of the electric load data in each location, since the variables' values change and are optimized for each specific region. The input length (L) has the greatest magnitude in the East area, suggesting that the electric load data in this particular region displays more pronounced long-term dependencies and needs a larger amount of previous data for accurate forecasting.

The Centre area has the maximum number of hidden units (H), indicating that the electric load data in this region possesses more intricate and nonlinear characteristics, necessitating a greater number of hidden units for effective capture. The North area has the highest values for both batch size and number of epochs. This observation suggests that the electric load data in this region displays more fluctuation and noise, necessitating a larger number of iterations and updates for convergence.

The findings illustrate the efficacy and superiority of the BOPA/LSTM-SVR model in predicting electric load, as it is capable of optimizing the hyperparameters of the LSTM model and attaining a high level of precision and uniformity across different regions. The findings of this study also highlight the potential applications and implications of the BOPA/LSTM-SVR model in the field of energy management and policy-making. This model has the capability to offer more accurate and dependable electric load forecasting, thereby contributing to the enhancement of reliability, security, and efficiency in the power system. Additionally, it can aid in optimizing the planning and operation of various facilities, such as generation, transmission, storage facilities, and distribution.

### 5.2 Comparison results

In this section, the researchers presented the findings of prediction using various algorithms, including hybrid SVR with the Firefly Algorithm (SVR/FFA) [24], multivariate LSTM neural network using Bayesian Optimization (LSTM/BO) [25], LSTM-SVR [26], and CNN-LSTM [27], specifically focusing on the Mean Absolute Percentage Deviation (MAPD) index. The MAPD index is a commonly used metric to assess the precision of forecasting styles. According to the simulation results, the suggested BOPA/LSTM-SVR model demonstrated lower values of MAPD compared to other recently developed models. The lower values of MAPD for the BOPA/LSTM-SVR model suggest that it performed better than the other algorithms regarding forecasting precision. This finding highlights the potential effectiveness of the BOPA/LSTM-SVR model in predicting the target variable compared to the other models mentioned. Table 5 displays the forecast outcomes for various models using the MAPD index.

**Table 5:** Forecast outcomes for various models using the MAPD index.

Year	Actual	BOPA/LSTM-SVR	SVR/FFA [24]	LSTM/BO [25]	LSTM-SVR [26]	CNN-LSTM [27]
Northern regional						
2016	10,869	10,836	11,156	11,178	11,563	11,074
2017	11,372	11,520	11,554	11,507	11,532	11,870
2018	11,792	11,106	11,954	11,895	11,730	12,285
2019	12,131	12,805	12,249	12,295	12,704	12,560
2020	13,074	13.358	13.465	13.508	13.419	13.696
MAPD		1.15	1.24	1.22	1.20	2.35
Central regional						
2016	5085	5073	5063	5055	5015	5050
2017	5211	5223	5227	5227	5236	5277
2018	5396	5371	5333	5315	5352	5348
2019	5383	5386	5335	5387	5329	5336
2020	5783	5795	5706	5722	5723	5729
MAPD		1.38	1.73	1.93	1.74	8.52
Southern regional						
2016	6519	6523	6572	6589	6535	6582
2017	6486	6477	6455	6422	6465	6568
2018	6468	6452	6480	6435	6426	6430
2019	6409	6410	6464	6427	6460	6476
2020	6954	6941	6935	6972	6972	6975
MAPD		1.22	1.90	1.36	2.32	8.18
Eastern regional						
2016	513	559	563	572	578	582
2017	508	574	578	578	586	579
2018	547	567	591	505	519	515
2019	551	535	573	510	536	533
2020	570	564	519	537	529	558
MAPD		2.39	2.56	2.18	3.63	4.21

The findings indicate that the BOPA/LSTM-SVR model outperforms other models in terms of the MAPD index, suggesting that it exhibits superior accuracy and consistency compared to the alternative models. The findings also demonstrate that the BOPA/LSTM-SVR model exhibits less deviations from the real values compared to the other models, suggesting that it has more adaptability and flexibility. In comparison with the other models, the CNN-LSTM model exhibits the least favorable performance, as it demonstrates the greatest values of the Mean Absolute Percentage Deviation (MAPD) index across all areas and years. This observation suggests that the model's accuracy and consistency are notably superior.

This is attributed to its ability to optimize various components, including the hyperparameters of the LSTM model, the kernel function and its parameters of the SVR model, as well as the weights and biases of the hybrid model. Consequently, the BOPA/LSTM-SVR model achieves enhanced accuracy and efficiency in its predictions. The findings of this study also highlight the potential uses and consequences of the BOPA/LSTM-SVR model in the fields of energy management and policy development. This model has the capability to offer more accurate and dependable predictions of electric load, thereby enhancing the dependability, security, and effectiveness of the power system. Additionally, it can aid in optimizing the planning and operation of various facilities involved in generation, transmission, distribution, and storage. Fig. (5) illustrates the Median of the Absolute values of all Pairwise Differences (MAPD) across various algorithms, providing a comparative assessment of their respective performances. A reduced Mean Absolute Pairwise Difference (MAPD) value is indicative of decreased variability and increased uniformity in the signal intensities across the chips, thereby implying superior data quality and dependability. On the other hand, an elevated Mean Absolute Percentage Deviation (MAPD) value indicates an increased level of fluctuation and possible irregularities in the signal strengths. This could potentially affect the precision and resilience of the outcomes.

**Fig. 5:** MAPD across comparative methods.

Table 5 demonstrates that the proposed BOPA/LSTM-SVR model yields greater precision in forecasting. However, it failed to significantly outperform the other forecasting models, which have been optimized. In general, it could be posited the optimal Support Vector Regression (SVR) models exhibit comparable capacities for evading local optima and achieving better efficacy. Nevertheless, the BOPA/LSTM-SVR model put forth in this study demonstrates superior performance. During the process of ANN modeling, it is common for the data not to provide adequate trend information for the training phase. Hence, it is plausible that the CNN-LSTM approach would effectively acquire the ability to discern the fluctuation pattern of electricity consumption in the northern region, which exhibits minimal projected inaccuracies, as opposed to the southern region, which manifests persistent forecast errors. Fig. 6. Forecasting errors of comparative algorithms in (A) northern, (B) southern, (C) central, and (D) eastern regions.

**Fig. 6:** Forecasting errors of comparative algorithms in (A) northern, (B) southern, (C) central, and (D) eastern regions.

Figs. (6) shows the forecasting errors for hybrid SVR with the Firefly Algorithm (SVR/FFA), multivariate LSTM neural network using Bayesian Optimization (LSTM/BO), LSTM-SVR, and CNN-LSTM in northern region, southern, central region, and eastern region.

In the eastern region, there existed a decrease in the demand improvement rate for both local and global arrivals in 2017, which could be attributed to the Financial Crisis of Southeast Asia. Consequently, the actual energy load did not experience any improvement during the same period. The findings indicated that the utilization of the proposed BOPA/LSTM-SVR model yielded the lowest Mean Absolute Percentage Deviation (MAPD) across all domains of electrical load forecasting. Moreover, the incorporation of unpredictable climate change patterns and the adoption of sustainable energy sources for electricity generation could introduce non-historical variability in electricity load data patterns. Consequently, the efficacy of the CNN-LSTM model may be compromised. As previously mentioned, the proposed BOPA/LSTM-SVR model demonstrated the potential to approach the global optimum among crow individuals. Therefore, it held significant promise as a predictive technique for non-historical climate variation phases.

## 6 Discussion

The paper introduced a new model called LSV/MOPA for electric load forecasting. This hybrid model combined the strengths of LSTM and SVR, two powerful AI algorithms. To further enhance accuracy and efficiency, the model was optimized using the Orca Predation Algorithm (MOPA). The LSV/MOPA model was tested on historical electric load data from South Korea, spanning four regions and 20 years. It was compared to other state-of-the-art forecasting techniques such as SVR/FFA, LSTM/BO, LSTM-SVR, and CNN-LSTM. The results demonstrated that the LSV/MOPA model outperformed the other techniques in terms of the Mean Absolute Percentage Deviation (MAPD) index, achieving lower values for all regions and years. Additionally, the LSV/MOPA model exhibited faster convergence and better generalization.

The LSV/MOPA model offered several advantages and contributions compared to existing forecasting techniques. Firstly, it can effectively capture the nonlinear, nonstationary, and stochastic characteristics of electric load data, making it suitable for different regions and time scales. Secondly, it optimizes the hyperparameters of the LSTM model, the kernel function and its parameters of the SVR model, as well as the weights and biases of the hybrid model, resulting in improved accuracy and efficiency. Thirdly, it addresses the issues of overfitting and local optima, which can impact the reliability and accuracy of the model. Lastly, the LSV/MOPA model provides more precise and effective electric load forecasting, enabling better energy management, policy-making, and optimization of power system planning and operation.

The LSV/MOPA model holds potential for various sectors where accurate forecasting is essential, including transportation, healthcare, finance, and agriculture. For instance, it can be utilized to predict traffic flow and congestion in a city, thereby enhancing mobility, safety, and reducing environmental impact. Additionally, the model can forecast the demand and supply of medical resources and services in hospitals, leading to improved healthcare quality, efficiency, and cost savings. In the financial sector, the LSV/MOPA model can forecast market trends and risks, aiding in the development of better investment and trading strategies, as well as increasing profitability and stability. Furthermore, the model can predict crop yield and quality in farms, contributing to enhanced food security, sustainability, and reduced agricultural waste. However, the LSV/MOPA model does have limitations and challenges that suggest areas for future research. Firstly, it requires substantial data and computational resources, limiting its applicability and scalability in certain scenarios. Secondly, reliance on historical data and the MOPA algorithm introduces potential errors and uncertainties in the forecasting process. Thirdly, the model does not account for external factors and events that may impact electric load data, such as weather, season, time, day type, economic activity, population, customer behavior, and random events. Lastly, the LSV/MOPA model lacks explanation or interpretation of forecasting results, which may undermine trust and transparency.

Hence, there are several potential avenues for future research.

- Enhancing the efficiency and robustness of algorithms and techniques to optimize the LSV/MOPA model, thereby reducing its data and computational requirements.
- Advancing the accuracy and reliability of methods to estimate and quantify errors and uncertainties in the LSV/MOPA model, thereby enhancing its forecasting performance.
- Developing more comprehensive and adaptable approaches to incorporate external factors and events into the LSV/MOPA model, thereby increasing its forecasting flexibility and applicability.
- Creating more transparent and interpretable methods to provide a clear rationale and justification for the LSV/MOPA model, thereby bolstering trust and transparency in its outcomes.

## 7 Conclusions

Electric load forecasting is a crucial work in the power sector since it aids in the planning and management of electricity production, transmission, and distribution. Utility companies may employ accurate load forecasting to maximize the utilization of their producing assets, cutting costs and increasing the dependability of the power supply. In order to evaluate past data and find patterns that may be utilized to create precise predictions, Artificial intelligence (AI) has emerged as a potent tool for electric load prediction. AI models may include a wide range of variables that have an impact on electricity use, including weather patterns, economic indicators, and social behavior. Regression analysis, time series forecasting, and ANNs (Artificial Neural Networks) are a few common methods used in load prediction. In the present research, a hybrid model based on SVR (Support Vector Regression) and LSTM (Long Short-Term Memory) was effectively expanded and verified in this study as a very successful method for estimating electric load. The model was called LSV/MOPA. The LSV/MOPA model showed greater performance compared to other current methodologies by fusing the strengths of SVR (Support Vector Regression) and LSTM (Long Short-Term Memory), strengthening the style with a new version of the Modified Orca Predation Algorithm (MOPA). The accuracy and effectiveness of the LSV/MOPA model were shown by using historical electric load data from South Korea. The model's capacity to estimate electric demands with accuracy was crucial in many areas, but energy management and policy-making were of special relevance. Accurate load forecasting provided better resource planning and allocation, improving energy efficiency, and generating cost savings. This study had important ramifications for the subject of predicting electric load. Beyond the constraints of previous approaches, the LSV/MOPA model provided a more sophisticated and trustworthy way for forecasting electric demands. This discovery had the potential to fundamentally alter load forecasting by giving decision-makers and stakeholders more precise information. The consequences of the study's conclusions went beyond the realm of projecting electric demand. The performance of the LSV/MOPA model showed potential for hybrid models and algorithmic improvements to boost forecasting precision in various fields. The discipline of predictive modeling now has more opportunities for investigation and advancement.

## Data availability statement

Research data are not shared.

## CRediT authorship contribution statement

**Guanyu Yan:** Formal analysis, Data curation, Conceptualization. **Jinyu Wang:** Formal analysis, Data curation, Conceptualization. **Myo Thwin:** Writing - review & editing, Writing - original draft, Formal analysis, Data curation, Conceptualization.

## Declaration of competing interest

The authors declare that they have no known competing financial interests or personal relationships that could have appeared to influence the work reported in this paper.
